The article "Impaired immunomodulatory capacity in adipose tissue‐derived mesenchymal stem/stromal cells isolated from obese patients" was published in 2021. Journal: J Cell Mol Med.

# Impaired immunomodulatory capacity in adipose tissue‐derived mesenchymal stem/stromal cells isolated from obese patients

**DOI:** 10.1111/jcmm.16869

**Published:** 2021-08-21

**Authors:** Xiang‐Yang Zhu, Nattawat Klomjit, Sabena M. Conley, Megan M. Ostlie, Kyra L. Jordan, Amir Lerman, Lilach O. Lerman

**Affiliations:** ^1^ Division of Nephrology & Hypertension Mayo Clinic Rochester MN USA; ^2^ Department of Cardiovascular Diseases Mayo Clinic Rochester MN USA

**Keywords:** inflammation, macrophage, mesenchymal stem cells, renal artery stenosis

## Abstract

Immune‐modulatory properties of adipose tissue‐derived mesenchymal stem/stromal cells (MSCs) might be susceptible to metabolic disturbances. We hypothesized that the immune‐modulatory function of MSCs might be blunted in obese human subjects. MSCs were collected from abdominal subcutaneous fat of obese and lean subjects during bariatric or kidney donation surgeries, respectively. MSCs were co‐cultured in vitro for 24 h with M1 macrophages, which were determined as M1or M2 phenotypes by flow cytometry, and cytokines measured in conditioned media. In vivo, lean or obese MSCs (5 × 10^5^), or PBS, were injected into mice two weeks after unilateral renal artery stenosis (RAS) or sham surgeries (*n* = 6 each). Fourteen days later, kidneys were harvested and stained with M1 or M2 markers. Lean MSCs decreased macrophages M1 marker intensity, which remained elevated in macrophages co‐cultured with obese MSCs. TNF‐α levels were four‐fold higher in conditioned media collected from obese than from lean MSCs. RAS mouse kidneys were shrunk and showed increased M1 macrophage numbers and inflammatory cytokine expression compared with normal kidneys. Lean MSCs decreased M1 macrophages, M1/M2 ratio and inflammation in RAS kidneys, whereas obese MSCs did not. MSCs isolated from lean human subjects decrease inflammatory M1 macrophages both in vivo and in vitro, an immune‐modulatory function which is blunted in MSCs isolated from obese subjects.

## 1 INTRODUCTION

Mesenchymal stem/stromal cells (MSCs) are derived from different adult (adipose tissue, peripheral blood, bone marrow) and neonatal tissues. MSCs are considered favourable candidates for regenerative medicine, given their numerous proangiogenic, anti‐inflammatory and antifibrotic activities achieved by paracrine mechanisms.^1^ We have previously shown that autologous MSCs infusion improves renal function in swine renal artery stenosis (RAS) and attenuates renal inflammation by decreasing macrophage accumulation.^2^, ^3^, ^4^, ^5^ Furthermore, adipose tissue‐derived MSCs express only low levels of MHC class‐I, and lack the major MHC class‐II molecules,^6^ allowing them to evade immune recognition. Thus, exogenously delivered MSCs can modulate the host immune response. The mechanisms involved in their immunomodulatory effects have not been fully elucidated and may depend on both cell contact‐dependent mechanisms and paracrine effects through production of cytokines and various soluble factors that regulate immune cell functions.^7^, ^8^, ^9^ Previous studies^10^, ^11^ demonstrated in vitro that healthy MSCs inhibit adhesion and invasion of inflammatory cells and promote polarization of macrophages from an inflammatory (M1) to anti‐inflammatory (M2) phenotype. Furthermore, adipose tissue‐derived MSCs exhibit advantageous capabilities in polarization of M1 macrophages and anti‐inflammatory effects compared to bone marrow‐derived MSCs.^12^

Obesity induces metabolic dysregulation including hyperglycaemia, hyperinsulinemia and dyslipidaemia, which are major risk factors for diabetes and cardiovascular complications. Shree et al.^13^ showed that injection of healthy human adipose tissue‐derived MSCs exerts beneficial effects in high‐fat diet‐fed mice. Moreover, obesity can trigger an early senescence programme in human adipose tissue‐derived MSCs, which exhibit lower proliferative capacities than non‐obese MSCs, suggesting impaired function.^14^ However, whether obesity affects the immunomodulatory capability of MSCs is unknown.

This study was therefore designed to test the hypothesis that MSCs from obese human subjects have impaired capability to reverse inflammatory macrophage phenotypes. To this end, we exposed macrophages to ‘lean’ or ‘obese’ human MSCs both in vitro and in a RAS mouse model in vivo.

## 2 METHODS

To evaluate the effects of obesity on their immunomodulation capacity, MSCs were obtained from human subjects with obesity and from lean controls, injected into mice with unilateral RAS, and renal macrophage phenotypes and spleen monocyte reservoir then determined 2 weeks after injection. Furthermore, to compare their direct impact on macrophages, obese and lean MSCs were co‐cultured with activated macrophages, and their phenotypes and cytokine release were determined.

### 2.1 Human subject recruitment and MSCs isolation

All human study procedures were approved by the Mayo Clinic Institutional Review Board. Eligible subjects were 18–80 years of age with a BMI < 30 kg/m^2^ (lean) or BMI > 35 kg/m^2^ (obese), who underwent kidney donor nephrectomy or weight reduction gastric surgery, respectively (*n* = 6 each), at Mayo Clinic in Rochester, Minnesota, between October 2017 and March 2019. All subjects gave written informed consent. Blood samples and body weights were collected prior to surgery. At the time of their surgical procedures, adipose tissue (0.5–2.0 g) samples were harvested and MSCs isolated following standard protocols.^2^, ^3^, ^4^, ^14^ Briefly, adipose tissue was minced, incubated with collagenase‐H at 37°C for 45 min, and after stopping, digestion was filtered through a 100‐μm cell strainer. The cellular suspension was centrifuged for 10 min at 233 *g* to pull down cells, and the cellular pellet re‐suspended in Advanced Minimum Essential Medium supplemented with 5% platelet lysate (PLTmax, Mill Creek Life Sciences). MSCs were then expanded in culture for three passages to prepare for experimentation.

Third‐passage MSCs (from both lean and obese subjects) were characterized by imaging flow cytometry (FlowSight, Amnis) to confirm expression of MSC‐specific surface markers CD73 (10 μl/10^6^ cells), CD90 (4 μl/10^6^ cells) and CD105 (20 μl/10^6^ cells), and rule out expression of CD45 (0.2 μl/10^6^ cells) (all from Abcam) or CD34 (20 μl/10^6^ cells, BD BioScience). We have recently confirmed that these MSCs were able to differentiate into adipocyte, osteocyte and chondrocyte lineages,^2^, ^3^, ^4^, ^14^ underscoring their mesenchymal lineage and that these properties were comparable between lean and obese MSCs.^14^ Culture media collected from both lean and obese MSCs were subsequently tested for levels of interferon‐γ, interleukin (IL)‐1a, IL‐6, IL‐10, monocyte chemoattractant protein (MCP)‐1, TNF‐α and the immunomodulatory factors indoleamine 2, 3‐dioxygenase (IDO)‐1 and prostaglandin‐E2 (PGE2) using ELISA.

### 2.2 In vivo study

To investigate the effects of obesity on the ability of MSCs to modulate macrophage phenotype in vivo, MSCs obtained from either lean or obese subjects (*n* = 6 each) were injected in mice with unilateral RAS. Kidney M1 and M2 macrophages were counted ex vivo in kidneys harvested 2 weeks after injection. Male 129–S1 mice (Jackson Laboratory) were studied for 4 weeks after induction of unilateral RAS or sham surgery at 11 weeks of age. Mice were randomly divided into sham, RAS+ vehicle, RAS+ lean MSCs and RAS+ obese MSCs (*n* = 6 each). All protocols were approved by the Mayo Clinic Institutional Animal Care and Use Committee.

Renal artery stenosis was induced by surgical placement of a 0.15 mm diameter arterial cuff, whereas sham surgeries without cuff placement were performed in the control group, as previously described.^5^, ^15^ After 2 weeks, the carotid artery was cannulated, and 200 µl phosphate‐buffered solution (PBS) or MSCs (5 × 10^5^ cells in 200 µl PBS, pre‐labelled with Far‐red dye) was slowly injected into the aorta. Two weeks later, the mice were euthanized with CO_2_. Kidneys were collected for ex vivo studies and weighed. Frozen kidney sections were stained with CD3 (1:100, Abcam) to evaluate rejection, and MSCs were counted per field to assess retention. Paraffin‐embedded kidney sections were stained with F4/80 (1:100, Abcam)/iNOS (1:100, Santa Cruz Biotech) for M1, F4/80 and mannose receptor‐1 (1:100, Abcam) for M2 macrophages. Ten images of each kidney section were taken with Zeiss microscope, and the number of M1 (F4/80^+^/iNOS^+^) and M2 macrophages (F4/80^+^/mannose receptor‐1^+^) was manually counted by double‐positive staining per field (20×). Furthermore, kidney gene expression of the inflammatory cytokines TNF‐α, IL‐6, IL‐1a and MCP‐1 was evaluated using qPCR.

### 2.3 In vitro macrophages study

To investigate the direct effects of obesity on the ability of MSCs to modulate macrophage phenotype in vitro, MSCs obtained from either lean or obese subjects were co‐cultured with M1 macrophages, and the M1/M2 phenotypes were subsequently determined. To generate M1 macrophages, human monocytes (U937 cells, ATCC, CRL‐1593.2™) were cultured in RPMI‐1640 supplemented with 10% FBS, 1% penicillin and streptomycin at 37°C in 5% CO_2_. Macrophages (M0) were induced by adding 100ng/ml phorbol 12‐myristate 13‐acetate (PMA, Sigma MO) for 12h. Then, classical activation models of M1 macrophages in vitro were established by treating M0 cells with 100 U/ml interferon (IFN)‐γ (R&D Systems, MN) and 5ng/mL lipopolysaccharide (LPS, Sigma, MO) for 24 h.^11^

The macrophages were then randomly divided into several groups: M0, M1, M1+Lean MSCs and M1+obese MSCs. Co‐culture was done using transwell (Costar polycarbonate filters, 5 μm pores), with macrophages seeded at the bottom chamber and MSCs added to the up chamber. We used a 24‐well transwell plate for imaging and a 6‐well transwell plate to collect macrophages for Western blotting, flow cytometry and culture media for ELISA. After a 24‐h co‐culture, M1 and M2 macrophages were phenotyped by both immunostaining and flow cytometry. F4/80^+^ (1:25, Abnova) and iNOS^+^ (1:100) M1, and F4/80^+^/mannose receptor‐1^+^ (1:100) M2 macrophage phenotypes were determined by immunofluorescence. Images were taken with Zeiss microscope, and M1 and M2 macrophage intensities were quantified using Zeiss Zen2 software. For flow cytometry, CD86 and CD64 were stained to detect M1, and CD163 and CD200R for M2 (all from BioLegend, 5 ul per test/10^6^ cells). These antibodies were selected based on their suitability for flow cytometry, as previously reported.^16^ At least 10000 events were counted, and the percentages of double‐positive CD64/CD86 (M1) and CD163/CD200R (M2) cells were determined. In addition, macrophages (M0, M1, M1+Lean MSCs and M1+obese MSCs) and their culture media were collected. Arginase‐1 expression in macrophages was then evaluated using Western blotting, and levels of IL‐1ra and TNF‐α in culture media using ELISA. ^16^

### 2.4 Statistical analysis

Results of normally distributed data are expressed as mean ± SEM and non‐normally distributed as median(Range). Comparisons within groups were performed using the paired Student's *t*‐test or Wilcoxon/Kruskal–Wallis test, depending on normality of distribution, and among groups using ANOVA and unpaired *t*‐test. Chi‐square or Fisher's exact tests were used for categorical variables analysis. A statistical difference was considered significant for *p *≤ 0.05.

## 3 RESULTS

Lean and obese subjects were of a similar age, but there were more women in the obese than in the lean group, BMI was higher (*p *< 0.001), and a history of hyperlipidaemia and diabetes was significantly more common in the obese group. As for medications, statins were primarily prescribed for hyperlipidaemia and metformin or glipizide for diabetes. The history of hypertension or the use of angiotensin‐converting enzyme inhibitors or calcium blockers was not different between lean and obese subjects. Furthermore, obese subjects had increased triglyceride and haemoglobin A1c levels, reflecting metabolic alterations in these subjects, although glucose levels were unchanged (Table 1).

**TABLE 1:** The demographics of lean and obese subjects (*n* = 6 each)

	Lean	Obese
Demographics		
Age (years)	56.6 ± 2.2	57.0 ± 2.6
Gender (female, %)	66%	83%
BMI (kg/m^2^)	29.1 ± 0.9	42.9 ± 1.1*
Medical history (% of patients)		
Hypertension	33%	50%
Hyperlipidaemia	18%	66%*
Diabetes	12%	66%*
Medications (% of patients)		
ACE inhibitors/Calcium channel blockers	33%	33%
Statins	6%	18%*
Metformin/glipizide	0%	33%*
Cholesterol (mg/dl)	184.4 ± 5.8	203.7 ± 25.9
Triglyceride(mg/dl)	95.4 ± 8.8	146.7 ± 25.3*
Glucose (mg/dl)	106.2 ± 5.9	125.4 ± 12.3
Haemoglobin A1c(mmol/ml)	5.3 ± 0.1	6.5 ± 0.4*

Abbreviations: ACE, angiotensin‐converting enzyme; BMI, body mass index.

* *p *< 0.05 vs. lean.

### 3.1 MSC characterization

Flow cytometry analysis showed that MSCs from both lean and obese subjects express CD73, CD90 and CD105 (purity 96.7%–99%) and were negative to CD45 and CD34 (Figure 1A), confirming their MSC nature.

**FIGURE 1:** MSCs surface markers, tracking and their effects on the kidney size in mice with renal artery stenosis. (A) Flow cytometry analysis and representative cell images show that human adipose tissue‐derived mesenchymal stem/stromal cells (MSCs) are positive for CD73, CD90 and CD105, but negative for CD45 and CD34. (B) Representative image showing no co‐localization of MSCs (red arrow) and CD3+ T lymphocytes (green arrow) in the stenotic mouse kidney. (C) The ratio of the stenotic and contralateral kidney weights was decreased in mice with renal artery stenosis (RAS) compared to sham and improved in mice injected with lean MSCs, but not with obese MSCs. *p < 0.05 vs. sham, ^#^ *p *< 0.05 vs. RAS

### 3.2 In vivo macrophage polarization

Mesenchymal stem cells retention rate in the kidney was not different between RAS+ lean and RAS+ obese (1.1 ± 0.6 vs. 0.7 ± 0.6 per field, *p *> 0.05) MSCs. No co‐localization of MSCs and CD3^+^ lymphocytes was observed, suggesting no immune rejection of human MSCs (Figure 1B). The weight ratio of stenotic/contralateral kidneys in RAS was significantly decreased in RAS+ vehicle, confirming renal atrophy. This ratio was slightly improved in RAS+ lean MSCs, but not in RAS+ obese MSCs (Figure 1C).

Renal artery stenosis kidneys showed an increase in both M1 (F4/80+/iNOS+) and M2 (F4/80+/mannose receptor‐1+) macrophage numbers and the M1/M2 ratio compared with normal mouse kidneys (Figure 2). RAS kidneys in mice treated with MSCs isolated from lean subjects showed decreased M1 macrophage numbers compared with RAS+ vehicle, whereas M1 macrophages remained high in RAS mice treated with obese MSCs. Similarly, MSCs isolated from lean subjects reversed M1/M2 ratio in RAS kidneys, which in RAS+ obese MSCs remained similar to RAS+ vehicle (Figure 2). Similarly, gene expressions of the M1‐related inflammatory cytokines TNF‐α, IL‐6, IL‐1a and MCP‐1 were all upregulated in RAS kidney, but significantly decreased in lean MSC‐treated groups (Figure 3A).

**FIGURE 2:** Lean but not obese MSCs reverse the macrophage inflammatory phenotypes in mice kidneys with renal artery stenosis. Representative images showing kidney interstitial macrophages in stenotic kidneys of mice treated with MSCs. Top: M1 macrophages (yellow arrow) double‐positive (yellow/orange when merged) for F4/80 (red) and iNOS (green). Middle: M2 macrophages double‐positive for F4/80 (red) and mannose receptor‐1 (green). Bottom: Image quantifications showed that stenotic RAS kidneys had increased numbers of M1 and M2 macrophages compared with sham. Compared with vehicle‐treated RAS, kidneys of RAS mice treated with MSCs isolated from lean subjects showed decreased M1 macrophage numbers and M1/M2 ratio, which remained elevated in RAS mice receiving obese MSCs. *p < 0.05 vs sham, ^#^ *p *< 0.05 vs. RAS

**FIGURE 3:** Lean MSCs downregulate the expression of inflammatory cytokines in vivo and reverse the macrophage inflammatory phenotypes in vitro (flow cytometry). (A) Gene expression of the inflammatory cytokines TNF‐α, IL‐6, IL‐1a and MCP‐1 increased in RAS compared to Sham kidneys. Lean MSCs downregulated their expression more effectively than obese MSCs. (B) Flow cytometry analysis showed that the numbers of in vitro stimulated M1 macrophages were decreased when co‐cultured with both MSC types, yet lean MSCs were more effective than obese MSCs. MSCs had no effects on M2 phenotype. *p < 0.05 vs. sham/M0, ^#^ *p *< 0.05 vs. RAS/M1, ^^^ *p *< 0.05 vs. lean MSCs

### 3.3 In vitro macrophage polarization

Flow cytometry demonstrated that in vitro, lean MSCs more effectively decreased M1 phenotype and M1/M2 ratio compared with obese MSCs (Figure 3B). Macrophages stimulated with IFNγ, and LPS showed increased CD68/iNOS intensity, indicating M1 induction. Co‐culture with lean MSCs decreased M1 intensity, which remained elevated in macrophages co‐cultured with obese MSCs (Figure 4). The downregulated arginase‐1 expression and increased release of TNF‐α levels by M1 macrophages were also consistent with phenotype switching, and MSCs reversed the switching. Importantly, lean MSCs were more effective in this respect (Figure 5A). Furthermore, the levels of IL‐1ra in cultured media decreased in M1, indicating decreased anti‐inflammatory potential, which were restored after MSC co‐culture, with lean MSCs more effective than obese MSCs. Also, M1 macrophages released more inflammatory cytokine TNF‐α, which decreased when co‐cultured with lean MSCs, but not with obese MSCs, partly due to greater TNF‐α release in obese MSCs (Figure 5A,B).

**FIGURE 4:** Lean MSCs decrease both M1 and M2 macrophage intensities while obese MSCs have the opposite effect when in co‐culture with M1 macrophages. Macrophages co‐cultured with MSCs isolated from lean subjects decreased both M1 (double‐positivity to CD68 in red and iNOS in green) and M2 (double‐positive to CD68 in red and mannose receptor‐1 in green intensity, while these remained high in macrophages co‐cultured with MSCs isolated from obese subjects. M1/M2 intensity ratios remained unaltered. *p < 0.05 vs. M0, ^#^ *p *< 0.05 vs. M1+obese MSCs

**FIGURE 5:** In vitro data show lean MSCs are superior to obese MSCs in their immunomodulatory capabilities. (A) Arginase‐1 protein expression in macrophages co‐cultured in vitro with MSCs isolated from lean or obese subjects, as well as IL‐1ra and TNF‐α levels in their culture media (*n* = 6 each). Lean MSCs blunted macrophage phenotype switching and immunomodulation‐associated cytokine release more robustly than obese MSCs. (*p < 0.05 vs. Lean or M0, ^#^ *p *< 0.05 vs. M1, ^^^ *p *< 0.05 vs. M1+lean MSCs). (B) Cytokine levels in the culture media of MSCs isolated from Lean and Obese subjects. IDO, indoleamine 2,3‐dioxygenase; IL, interleukin; INF, interferon; MCP, monocyte chemoattractant protein; PGE2, prostaglandin‐E2; TNF, tumour necrosis factor.*p<0.05 vs. lean

Levels of TNF‐α were higher in conditioned medium collected from obese MSCs than that from lean MSCs, whereas other cytokines tended to be elevated (*p *= 0.09), but did not reach statistical significance levels. Interestingly, levels of the immunosuppressive factor IDO‐1 were increased, whereas PGE2 decreased in obese MSCs (Figure 5B).

## 4 DISCUSSION

This study reveals that obesity impairs the capability of MSCs to transform macrophages towards an anti‐inflammatory phenotype both in vivo and in vitro. The immunomodulatory dysfunction of obese MSCs might in turn reflect attenuated tissue repair capacity and warrants interventions to support wound healing in obese subjects.

The adipose tissue represents a complex endocrine organ containing several different cellular populations, including adipocytes, MSCs and immune cells like macrophages and lymphocytes. We have previously^17^ demonstrated in obese pigs a shift towards amplified numbers of pro‐inflammatory macrophages and levels of the inflammatory cytokine TNF‐α in subcutaneous adipose tissue. This alteration promotes a chronic low‐grade inflammation and may negatively affect MSC progenitor function, hindering the ability of MSCs to support immunomodulatory function. This notion was supported by the current study showing impaired immunomodulatory capability in adipose tissue‐derived MSCs isolated from obese human subjects. These subjects not only had increased BMI but also increased circulating levels of triglycerides and haemoglobin A1c, indicating systemic metabolic alterations that may affect MSC function. Furthermore, obese MSCs exhibited significantly elevated release of the inflammatory cytokine TNF‐α into conditioned media, reflecting this pro‐inflammatory shift.

While many macrophage subsets exist, the two main classifications^18^ include classically activated, pro‐inflammatory M1 macrophage subtype, generated by exposure to LPS and IFN‐γ, which express iNOS, CD86 and CD64, and release IL‐1, IL‐6 and TNF‐a, and alternatively activated, anti‐inflammatory, presumably reparative M2 macrophage subtype, that are induced by IL‐4 and/or IL‐10 and express arginase‐1, mannose receptor‐1 (CD206), CD163 and CD200R. The ability to induce a change in macrophage phenotypes from an inflammatory M1 to anti‐inflammatory M2 is often associated with improved reparative function and blunted inflammation.

During acute or chronic kidney injury, molecular cross‐talk between the nephron epithelia and other cell types, including immune cells, regulates reparative responses.^19^ Immune cells like macrophages and dendritic cells have emerged as key players in the recovery of kidney function.^7^ This study confirms the immunomodulatory potency of MSCs reflected in their ability to switch macrophage phenotypes in vivo. The decrease in numbers of M1 macrophages in the RAS kidney by lean MSCs may reflect an overall decline in the inflammatory microenvironment in the kidney, which might benefit renal tissue repair. The impact of MSCs on immune or inflammatory disorders might derive from their paracrine effects, involving release of various soluble factors that regulate immune cell functions.^20^ The improvement of inflammatory milieu in lean compared to obese MSCs is translated into preserving renal tissue as reflected in decrease stenotic kidney atrophy and inflammatory cytokine expression.

Comparably, obese MSCs failed to decrease the numbers of M1 macrophage in vitro, possibly due to their greater release of the inflammatory cytokine TNF‐α, as detected in the culture medium. TNF‐α is an important mediator of macrophage polarization towards the inflammatory M1 phenotype.^21^ Furthermore, obese MSCs were less effective than lean MSCs in upregulating the anti‐inflammatory cytokine IL‐1ra in vitro when co‐cultured with M1 macrophages. Interestingly, obese MSCs released higher levels of immunosuppressive IDO‐1 and lower PGE2 compared to lean MSCs, possibly reflecting activation of compensatory mechanisms. Overall, these observations are consistent with altered immunomodulatory function in these cells. The observation that MSCs successfully alter macrophage phenotype in vitro lends credence to the stipulation that they might have a direct in vivo effect on M1 macrophages in situ. Moreover, the gap between lean and obese MSCs in their ability to switch M1/M2 ratio in vivo and in vitro suggests that the local microenvironment in injury sites may impact MSC function and thereby healing power.

Our study has several strengths, including comprehensive in vivo and in vitro studies of human MSCs. The use of statins^22^, ^23^ may enhance MSCs function in tissue repair, and metformin^24^ may enhance their immunomodulatory potential. Although obese individuals were more likely to be treated with these medications, their MSCs manifested inferior immunomodulatory functions than MSCs from lean individuals, implying overwhelming effects of obesity on MSC functions. Our control cohort was not truly ‘lean’, given that BMI 25–30 kg/m^2^ is considered ‘overweight’, but the mandated BMI gap of 5 kg/m^2^ ensured the separation of the groups. Furthermore, these subjects were eligible kidney donors screened for medical conditions and therefore relatively healthy subjects. Our small sample size may not have missed some small differences, and we studied only common macrophages populations. The image quality of macrophage staining in vitro was modest due to the use of a transwell, yet the staining colour, intensity and differences among the groups are clear. Moreover, we established macrophage polarization primarily using flow cytometry. We have also shown before that swine obesity modifies MSC cargo and impairs mitochondrial structure and functions,^25^, ^26^ all of which could potentially be linked to their interactions with inflammatory cells. Future studies are warranted to assess the direct mechanisms by which obesity or other metabolic conditions interfere with human MSC functions, as well as their ability to modulate other types of immune cells.

In summary, our study demonstrates that obesity impairs the ability of human MSCs to switch macrophage phenotype from M1 to M2 both in vitro and in vivo. Furthermore, obese MSCs may have altered ability to regulate circulating inflammatory monocytes by controlling monocyte reservoir in the spleen. The finding that MSCs from lean and relatively healthy subjects regulate monocytes and macrophages may provide a novel target for applying MSCs in diseases of immune dysfunction. Moreover, these observations also suggested attenuated capability of MSCs in obese patients to suppress inflammation and may contribute to impaired wound healing in these subjects.

## CONFLICTS OF INTEREST

Dr. Lerman is an advisor to AstraZeneca and Janssen Pharmaceuticals. The authors confirm that there are no conflicts of interest.

## AUTHOR CONTRIBUTIONS

**Xian‐Yang Zhu:** Conceptualization (lead); Data curation (lead); Formal analysis (lead); Methodology (lead); Writing‐original draft (lead). **Nattawat Klomjit:** Data curation (supporting); Writing‐review & editing (supporting). **Sabena Conley:** Data curation (supporting). **Megan M Ostlie:** Data curation (supporting); Formal analysis (supporting). **Kyra L. Jordan:** Data curation (supporting); Methodology (supporting). **Amir Lerman:** Writing‐review & editing (supporting). **Lilach Lerman:** Conceptualization (equal); Project administration (lead); Supervision (lead); Writing‐review & editing (supporting).

## Data Availability

Original data are available per request.
